The article "The Use of Infrared Thermography in Determining Timing for Early Pedicle Division of the Preexpanded Bipedicled Visor Flap after Ischemic Preconditioning" was published in 2022. Journal: Appl Bionics Biomech.

# The Use of Infrared Thermography in Determining Timing for Early Pedicle Division of the Preexpanded Bipedicled Visor Flap after Ischemic Preconditioning

**DOI:** 10.1155/2022/8564922

**Published:** 2022-07-26

**Authors:** Wentian Xiao, Shunuo Zhang, Hua Li, Shaoqing Feng, Fabio Nicoli, Richard Huynh, Jiajing Lu, Yixin Zhang, Peiru Min

**Affiliations:** ^1^Department of Plastic and Reconstructive Surgery, Shanghai Ninth People's Hospital Affiliated to Shanghai Jiao Tong University School of Medicine, Shanghai, China; ^2^Department of Plastic and Reconstructive Surgery, Royal Victoria Infirmary Hospital NHS Foundation Trust, Newcastle upon Tyne, UK; ^3^Department of Dermatology, Shanghai Skin Disease Hospital, School of Medicine, Tongji University, Shanghai, China

## Abstract

**Background:**

The preexpanded bipedicled visor flap, supported by the bilateral superficial temporal vessels, stands as an ideal choice for upper and lower lip reconstruction in males. However, the bilateral tissue bridges after flap transfer caused patients significant cosmetic deformity and psychological burden. Early division of bilateral pedicles reduced the length of hospitalization and expenses. In this study, infrared thermography (IRT) was used to guide the early pedicle division after ischemic preconditioning.

**Methods:**

This study retrospectively analyzed patients who underwent preexpanded bipedicled visor flap surgery from April 2018 to October 2021. Pedicle division was scheduled at two weeks postflap transfer. Ischemic preconditioning was initiated 3-5 days in advance by repeatedly clamping both pedicles. The temperature alteration of the flap and the temperature difference compared to the normal adjacent tissue were evaluated by IRT. The division surgery was not scheduled until the perfusion assessment indicated adequate. This comprised of subjective examination and indocyanine green angiography. The threshold of temperature difference to determine the pedicle division was analyzed based on the temperature changes between the clamps.

**Results:**

A total of 8 male patients successfully conducted the pedicle division without any complications. The delay period after ischemic preconditioning ranged from 14 to 19 days (average 16 days). Through ischemic preconditioning training, the average temperature of the flap gradually increased from 31.85 ± 0.36°C to 33.89 ± 0.50°C, and the temperature difference with the normal surrounding tissues decreased from 2.89 ± 0.30°C to 1.15 ± 0.46°C (95% confidence interval (1.5, 0.8)). The temperature difference stayed unchanged after pedicle division.

**Conclusion:**

Ischemic preconditioning shortens the perioperative period to pedicle division. Monitoring the temperature change reflects the revascularization between the flap and the recipient site, thus guiding the pedicle division. The temperature difference less than 1.5°C after clamping both pedicles can be set as the safe threshold for pedicle division.

## 1. Introduction

Defects of the upper and lower lip resulted from severe burns, trauma, or tumor resection seriously affect facial appearance and quality of life, and the reconstruction of such defects poses a great challenge for plastic surgeons [1]. For males, a potential option is the visor scalp flap. This technique was first described by Dufourmentel in 1919 [2] and is the ideal modality for lip reconstruction, especially for patients with severe burns. The visor scalp flap is supported by the bilateral superficial temporal vessels with robust blood supply, and this hair-bearing flap can also be used for facial beard reconstruction [3]. By utilizing tissue expansion technology, the donor site can be closed by primary intention [4].

Despite the advantages mentioned above, the clinical application of this technique has not been widely adopted for several reasons. Firstly, this flap usually requires a prolonged expansion period of 6 to 8 months. Secondly, it is a multistaged operative process with an unknown flap delay cycle, therefore a complicated postoperative care protocol was required to ensure success. Based on our previous experience, division of each pedicle should be performed at a 3-week interval to ensure flap survival [5]. This results in at least a 6-week perioperative period. During this period, the tissue bridges spanning the patient's tempus and facial-neck region cause severe facial deformity [6]. This presents great psychological and physical burden to the patient and increased the expense simultaneously.

By blocking part of the blood supply, a relatively low-oxygen tissue microenvironment promotes angiogenesis, thus accelerating the revascularization between the flap and recipient site, termed as ischemic preconditioning [7]. Ischemic preconditioning by clamping the pedicle shortens the interval required between pedicle divisions, reducing the flap delay cycle [8]. Rigorous evaluations of the revascularization status including clinical examination (color, swelling, and capillary reaction), laser Doppler flowmetry (LDF), and indocyanine green (ICG) angiography are required before pedicle division to ensure surgical outcome [9–12]. Clinical examinations are highly subjective based on surgeon's clinical experience. LDF assesses the perfusion by quantifying hemoglobin content in tissue but can be easily disrupted by movement and the cost is expensive. ICG angiography has been widely used as a modality to evaluate flap perfusion. However, ICG needs to be invasively injected and a quite considerable equipment is entailed. Due to the limitations of these devices, plastic surgeons are always searching for a safer, easy-to-use, and more reliable imaging device for evaluation.

Physiologically, perfusion affects tissue metabolism which in turn affects the tissue temperature [13]. Infrared thermography (IRT) monitors the temperature by detecting the infrared radiation emitted from tissue. Recently, it has gained popularity in plastic surgery, such as detecting the perforator preoperatively or evaluating the flap perfusion intra- and postoperatively [14–18].

To the best of our knowledge, the application of IRT for pedicle division has not been reported. In this study, IRT was applied in the early and one-time pedicle division of the preexpanded bipedicled visor flap after ischemic preconditioning. Clinical examination and ICG angiography were performed as criteria for safe detachment and the temperature changes during this period were recorded. This study was aimed at obtaining the safe threshold of temperature difference to determine the time for pedicle division.

## 2. Patients and Methods

### 2.1. General Information

This study retrospectively analyzed the patients suffering from severe burns on the upper and lower lips in a single center (The Shanghai Ninth People Hospital, Department of Plastic and Reconstructive Surgery) from April 2018 to October 2021. It was approved by the local ethics committee and followed the Helsinki Declaration. The study was considered exempt from registration since the data was collected retrospectively and the detecting methods were noninvasive. Fully informed consent and photographic authorization were obtained from all patients.

These patients received the preexpanded bipedicled scalp visor flap procedure for upper and lower lip reconstruction [5, 19]. A 500 ml to 800 ml tissue expander was implanted under the scalp and expanded to 2.5 to 3 times volume during a 6-month expansion period. The bipedicled visor flap was elevated by the same senior surgeon in a standard method as previously described in the literature. After the flap was transferred to resurface the defects on the upper and lower lips, the bilateral pedicles were exposed and covered with Vaseline gauze instead of skin grafting. This was performed to avoid secondary damage considering that the donor site for the necessary skin grafting was relatively rare and precious for burn patients. The disadvantage of this procedure was the exudation from the pedicle tissue requiring the gauze to be replaced regularly. The brief surgical procedure is shown in Figure 1.

### 2.2. Ischemic Preconditioning

Two weeks following flap transfer was chosen as the time point for pedicle division. Ischemic preconditioning was performed 3 days in advance. A rubber tube was wrapped around each pedicle of the flap and was tightened gradually to block the blood supply from the bilateral pedicles. A hand-held Doppler was used at the distal end of the pedicle to monitor the pulse of the superficial temporal artery to ensure the complete blocking. This protocol was carried out 3 times a day, and the clamping time was gradually extended from 30 min to 1 h according to the results of perfusion assessments.

### 2.3. Perfusion Assessments (Subjective Assessments, ICG, and IRT)

The hair on the flap was shaved daily to facilitate the perfusion assessment after clamping the pedicle. The regions of interest (ROIs) included the main part of the flap in the center for reconstruction, the suspended tissue bridge on both sides, and the normal surrounding tissue. Clinical examination of color change, degree of swelling, and the capillary reaction were assessed.

A hand-held thermal camera (FOTRIC® 228s, FOTRIC Inc., Shanghai) was performed at 50 cm from the midfacial region [15]. The palette was set in “Iron” mode and the temperature threshold was adjusted from 26°C to 36°C. The temperature readings of each ROI from the thermogram were obtained by the AnalyzIR software. To ensure adequate test and retest reliability in the temperature measurements, we applied a high-precision thermal camera with a thermal sensitivity of 0.03°C, and the whole process was carried out at the room with a central air conditioning system to maintain the room temperature at around 25°C. Temperature calibration with the environment was required before every test by routine.

When satisfactory signs from subjective assessments were elicited after pedicle clamping, the ICG angiography was conducted as a final check before pedicle division. The perfusion imaging of the patient's face and flap after ICG injection was monitored using an ICG device (PDE-NEO®II C10935-300, Hamamatsu Photonics, Hamamatsu-City), including both the arterial and venous phases. When the perfusion assessment indicated appropriate arterial supply and venous outflow, the operation of simultaneous pedicle division was scheduled.

### 2.4. Operation

The same senior surgeon performed all operations. The patient was anesthetized in the supine position, and IRT was used to record the stable temperature of the ROIs as the baseline when the patient was in stable anesthesia. One side of the pedicle was first detached, and the temperature was monitored. Then, the other pedicle was clamped to examine the color, swelling, capillary reaction, and temperature change. If the examination findings were satisfactory and no apparent temperature decrease was observed, the other pedicle was deemed ready to be separated. Otherwise, the flap was considered to have inadequate revascularization, and the other pedicle was reserved for the next operation. After both pedicle divisions, the temperature was recorded again. To summarize, IRT was used to record the tissue temperature before pedicle division, after one-side division, after clamping the other side, and after division on both sides. All results were measured when reaching the stable temperature (Figure 2).

### 2.5. Statistical Analysis

The temperature changes of all ROIs during the period from the first clamping training to the time when the blood supply was rated as satisfactory were recorded to summarize the temperature threshold to guide the safe pedicle division. The temperature value was expressed as $\overset{¯}{X}\pm \sigma$, and the paired 2-tailed *t* test was used to compare the mean temperature change between each ROI during the training period. Statistical analysis was performed using SPSS 22.0.

## 3. Results

A total of 8 male patients were included in this retrospective study for reconstruction of the upper and lower lips with the preexpanded bipedicled visor flap. All patients had severe burns on the middle and lower face. The patients were between 19 and 58 years old with an average age of 39 years. All patients successfully underwent pedicle division in one step without two-stage operation. The delay time of flap division after the first stage was from 14 to 19 days, with an average of 16 days. There were no related surgical complications or flap necrosis. After the pedicles were successfully divided, the subsequent flap trimming and laser hair removal treatment were arranged according to the patient's needs. The participants were satisfied with the outcomes of the cosmetic appearance (Figure 3).

We measured the temperature of each ROI (the main part of the flap, tissue bridges, and the surrounding normal tissue) before and after clamping the pedicle, and the temperature difference was calculated (Table 1). A typical process is shown in Figure 4. Prior to clamping the pedicle, all ROIs presented with a uniform temperature distribution. No significant temperature difference was observed. After the first clamping, the temperature differences of the flap and the tissue bridges between the surrounding normal tissues were 2.89 ± 0.30°C and 4.01 ± 0.48°C, respectively. At this point, the color of the flap became darker, showing signs of insufficient venous drainage (Figure 4(b), though not easy to distinguish from the photo due to the color of the scalp). When clamping the pedicle to the extent where the perfusion was identified as sufficient, the temperature of main body increased from 31.85 ± 0.36°C at the first clamping to 33.89 ± 0.50°C. The temperature difference between the main body and the surrounding normal tissue was 1.15 ± 0.46°C (95% confidence interval (1.5, 0.8)), while for the tissue bridges, the temperature difference was 3.60 ± 0.36°C with a statistical difference (*p* < 0.001).

Immediately after successful division, the temperature difference was 1.05 ± 0.59°C. Paired *t* tests confirmed no statistical difference (*p* = 0.48) between the postclamping and postdivision temperature difference. This result suggested the potential value of using the temperature difference after clamping to predict the postdivision flap perfusion.

## 4. Discussion

This study was aimed at applying IRT to evaluate the revascularization in the flap and determine the timing for pedicle division. We conducted that the ischemic preconditioning by repeatedly clamping the pedicle accelerated the revascularization process. We found that the temperature of the flap decreased significantly at the initial stage of the clamping training, indicating poor revascularization. As the ischemic preconditioning progressed, the temperature difference between the average temperature of the flap and the surrounding normal tissue gradually decreased from 2.89 ± 0.30°C to 1.15 ± 0.46°C, significantly lower than that of the suspended tissue bridge on both sides. This temperature change reflected the better revascularization between the flap and the recipient site during the ischemic preconditioning. Through repeated preconditioning, the hypoxic microenvironment in the tissue stimulated angiogenesis and promoted perfusion from the recipient area to the flap tissue [20, 21].

Through statistical analysis, we set the upper limit of the 95% confidence interval (95% CI) 1.5°C as the safety threshold for pedicle division. We also found that the postdivision temperature difference was consistent with the postclamping status. Therefore, by monitoring the postclamping temperature, perfusion patterns after pedicle division may be inferred to predict the surgical outcome.

Skin temperature is known to be actively determined by local metabolic processes, core heat transfer, and local tissue perfusion. There have been numerous studies investigating the use of IRT for evaluating tissue perfusion. Merla et al. established a biological heat conduction model of human tissue [22]. By comparing the results of IRT and LDF, they summarized the conversion relationship between these two methods and concluded that IRT was faster and more accurate in evaluating tissue perfusion. Sagaidachnyi et al. applied spectral filtering to process thermal image data [23]. The data showed a good correlation with the LDF results, and they concluded that IRT could be used as a tool for evaluating peripheral hemodynamics. In flap surgery, Weerd et al. applied dynamic IRT to assess the blood reperfusion of free flaps intraoperatively by observing the rewarming rate of the flap [24]. All these mentioned above indirectly reflected that the tissue perfusion could be embodied in the forms of temperature. We believe that both flap ischemia and congestion contribute to circulatory disorders, which leads to a temperature decrease because of the insufficient perfusion. Figures 4(c) and 4(d) demonstrated the signs of venous drainage disorder, and the thermogram showed obvious temperature dropping after pedicle clamping. For the flap ischemia, which may result from insufficient artery supply, studies have shown that temperature difference of more than 3°C could be noticed when the artery was compromised [25]. In this study, the revascularization process was presented by the gradual decrease of temperature difference after intermittent ischemic preconditioning. As the process of revascularization continued to mature, the perfusion ability from the wound base to the flap and the blood flow in the flap increased; thus, the temperature difference decreased.

In this study, we combined the subjective indicators of the flap and ICG angiography for perfusion evaluation. For certain particular flap types, such as the scalp flap we applied in this study, or flaps with dark complexion, the surgeon's judgment could be interfered. A typical case is shown in Figure 4(b), where the color change was not easily distinguished despite a significant temperature dropping and a prolonged capillary reaction time for the first clamping. ICG angiography stands for another common method for evaluating perfusion. By monitoring the relative perfusion rate of the flap compared to the normal adjacent tissue, the timing for pedicle division of the forehead flap could be advanced to 1-2 weeks postoperatively with careful evaluation of ICG angiography [26]. However, the application of ICG involves intravenous injection of indocyanine green; this process is considered as an invasive operation that needs an informed consent [12]. Repeated ICG angiography is likely to cause greater discomfort to the patient, and the equipment for ICG is cumbersome and quite expensive. On the contrary, IRT possessed a noninvasive detection process and can be applied repeatedly at any time, avoiding traumatic maneuvers and discomfort to the patient [27–29]. Furthermore, it can be universally applied with less interference due to skin color.

While the preexpanded bipedicled visor flap presents with an ideal method for reconstruction of upper and lower lip defects in males [5], this flap type has not been widely discussed or promoted clinically due to the complexity of the postoperative care process, the restricted application to male patients, and the obscure standard for pedicle division. The use of this flap involves long-term tissue expansion (approximately 6 months). Therefore, for safety reasons, in our previous experience, a more conservative surgical method of unilateral division with a 3-week interval was used to prevent flap necrosis out of insufficient perfusion, leading to the abandonment of all previous efforts. In this study, the ischemic preconditioning was performed to successfully shorten the division time (second stage) to 14-19 days under the temperature monitoring of the flap. This reduces the patient's perioperative discomfort and hospitalization costs [30, 31]. For safety concerns, we also applied IRT to prudently monitor the temperature change during the operation at each step. Once the flap encountered the sign of insufficient perfusion or a significant temperature dropping, we would retain the unilateral pedicle until the next operation. This safety precaution minimized the possibility of flap necrosis postoperatively.

In our opinion, this evaluation method can also be used in other types of pedicle flap or flap tube before the division, such as the forehead flap, the inguinal flap, or deltopectoral flap. Although the safe threshold for different flap types may be different, this study provided a practical modality to evaluate the revascularization process. The limit to this study is that the temperature of tissues is easily affected by factors such as the ambient temperature or whether the tissue itself encounters inflammation or infection. Therefore, we tried our best to ensure that the measuring environment was stable at about 25°C and excluded flaps with signs of infection or inflammation. In addition, clamping the pedicles for ischemic preconditioning brings inevitable pain to patients. Patients need to be fully informed before clamping process.

## 5. Conclusion

For preexpanded bipedicled visor flap, the ischemic preconditioning shortens the delay time. A temperature difference less than 1.5°C compared to the normal peripheral tissue can be set as the safe temperature threshold for pedicle division for this flap kind. Monitoring the temperature change of the postclamping flap reflects the perfusion of the flap and the revascularization with the recipient site as the postdivision temperature stays consistent with the postclamping temperature. IRT is portable and convenient to use for guiding the pedicle division.

## Figures and Tables

**Figure 1:** Surgical procedures of the preexpanded bipedicled visor flap. (a) Tissue expansion and flap design: a total volume of 800 ml was achieved for tissue expansion and the flap was designed based on the bilateral superficial temporal vessels. The red arrow indicated the running course of the superficial temporal vessel. (b) Flap harvest: the visor flap was elevated according to the flap design with the superficial temporal vessels intact as pedicles at the two sides. (c) Scar excision: the scar and periwound contraction of the lower lip and the anterior cervical region were thoroughly released. (d) Flap transfer: the elevated flap was rotated 180 degrees to cover the recipient site.

**Figure 2:** Monitoring of the temperature change during each stage of the operation (temperature threshold: 22-36°C). (a) The baseline temperature after stabilized anesthesia. (b) The temperature after the division of the left pedicle. (c) The temperature after clamping the right pedicle. (d) The temperature after both divisions. (e) The intraoperative flap appearance (the left pedicle was detached). Note that no obvious difference between the postclamping and the postdivision temperature of the flap.

**Figure 3:** (a–d) The patient's appearance before flap transfer with the tissue expander implanted and 6 months after pedicle division, respectively.

**Figure 4:** A typical process of temperature change (temperature threshold: 26-36°C). (a and b) The baseline appearance and temperature before the first clamping. (c and d) After the first clamping, the temperature dropped significantly and the color of the flap turned darker, although the color change was not easily recognized from the photo due to the color of the scalp. (e and f) After training for 4 days, the subjective evaluation was satisfied and the temperature of the main body showed narrowed decline, while the temperature of the tissue bridge still dropped significantly. (g and h) ICG angiography: (above) the perfusion originated from the recipient site and (down) the whole main body of the flap was perfused well and the perfusion to the tissue bridge was insufficient.

**Table 1:** Temperature measured with infrared thermography.

Patient no.	First clamping			Clamping to satisfied perfusion			After pedicle division	
	Tissue bridge	Flap	Surrounding	Tissue bridge	Flap	Surrounding	Flap	Surrounding
1	30.7	32	34.9	31.2	34	34.5	34.3	34.5
2	30.5	31.8	34.6	31	33.8	34.9	33.7	34.1
3	29.7	31.5	34.2	30.5	33.2	34.4	33.6	34.5
4	31	32.2	35.6	31.8	34.3	35.8	34.4	36
5	31.1	32.5	34.9	32.1	34.8	35.2	34.5	35.3
6	31	31.5	34.7	31.6	33.4	35	34.2	36
7	30.4	31.7	34.5	31.5	33.9	35.4	33.8	34.9
8	31.4	31.6	34.5	31.8	33.7	35.1	33.6	35.2
Average temperature	30.73 ± 0.53	31.85 ± 0.36		31.44 ± 0.52	33.89 ± 0.50		34.01 ± 0.38	35.06 ± 0.70
Temperature difference	4.01 ± 0.48	2.89 ± 0.30		3.60 ± 0.36	1.15 ± 0.46		1.05 ± 0.59	

## Data Availability

All data used to support the findings of this study are included within the article.
